The article "Bone Cancer Detection Using Feature Extraction Based Machine Learning Model" was published in 2021. Journal: Comput Math Methods Med.

# Bone Cancer Detection Using Feature Extraction Based Machine Learning Model

**DOI:** 10.1155/2021/7433186

**Published:** 2021-12-20

**Authors:** Ashish Sharma, Dhirendra P. Yadav, Hitendra Garg, Mukesh Kumar, Bhisham Sharma, Deepika Koundal

**Affiliations:** ^1^Department of Computer Engineering & Applications, GLA University, NH#2, Delhi Mathura Highway, Post Ajhai, Mathura, (UP), India; ^2^Chitkara University School of Engineering and Technology, Chitkara University, Himachal Pradesh, India; ^3^School of Computer Science, University of Petroleum & Energy Studies, Dehradun, India

## Abstract

Bone cancer is considered a serious health problem, and, in many cases, it causes patient death. The X-ray, MRI, or CT-scan image is used by doctors to identify bone cancer. The manual process is time-consuming and required expertise in that field. Therefore, it is necessary to develop an automated system to classify and identify the cancerous bone and the healthy bone. The texture of a cancer bone is different compared to a healthy bone in the affected region. But in the dataset, several images of cancer and healthy bone are having similar morphological characteristics. This makes it difficult to categorize them. To tackle this problem, we first find the best suitable edge detection algorithm after that two feature sets one with hog and another without hog are prepared. To test the efficiency of these feature sets, two machine learning models, support vector machine (SVM) and the Random forest, are utilized. The features set with hog perform considerably better on these models. Also, the SVM model trained with hog feature set provides an *F*1-score of 0.92 better than Random forest *F*1-score 0.77.

## 1. Introduction

A human body consists of 206 bones. Bones are attached to the muscle of the body and provide support for the movements. Bone ligaments are fibrous tissue and filled with spongy bone marrow. A bone cancer originates from the healthy cells and starts forming a tumor (Blackledge et al. 2014) [1]. The primary symptom of bone cancer is a bone tumor. The tumor grows gradually and may spread to the other part of the body. It can destroy the bone tissue and bone becomes weaker. According to statics, 3500 people in the United State were affected by bone cancer in the year 2018, and approx. 47% of the bone-cancer diagnosed people died. The doctor diagnoses cancer via many tests. The X-ray image diagnosis is used to detect cancer in the human bone. The healthy bone and the cancerous bone X-ray assimilation rates are different. Due to which a cancerous bone image surface appears ragged (Oishila et al. (2018) [2]). The bone cancer severity is measured by a stage and the grade. Tumor (geographic bone destruction) growth rate is used by doctors to predict the disease growth rate. Diagnosing cancer in the bone requires expertise. Bone cancer diagnoses are performed manually by a doctor, so it may take time, and error possibility arises.

Early detection seems to be the only factor that increases the chance of survival of cancer-affected patients. This paper deals with the system which uses the machine learning algorithm SVM and image processing techniques to detect the tumor and classify cancer. Similar researches in this field have been carried out by researchers to develop an automated system to assist a doctor. An automated system is fast with low error probability. Machine learning algorithm SVM and digital image processing technique, preprocessing, edge detection, and feature extraction have been used to develop an automated system (Chen et al. 2007) [3]. In the other research, Yadav and Rathor (2020) [4] developed an automated system for the diagnosis of human bone. They have utilized a deep neural network to categorize healthy and fracture bone. The model is trained with the large volume of the augmented image dataset. In the augmentation process, the same copy of images is generated which may be present in the training and test dataset. A *k*-fold cross-validation can be used to avoid bias performance.

Asuntha and Srinivasan (2017) [5] have used the GLCM feature to identify fractured bone. In the experiment, they concluded only GLCM-based texture feature is not sufficient to correctly identify the cancerous bone. The entropy and skewness also play a vital role in cancerous region prediction. The value of entropy is low in the cancerous region and high outside the cancerous region. The hog feature gives the shape and direction of a pixel in images. Bandyopadhyay et al. (2018) [2] have used a fusion of several techniques and texture features to identify and classify the cancerous bone and the healthy bone. The classification of the long bone is performed using SVM. The method is focused only on the long healthy and cancerous bone. The performance of models is 85%, which can be further improved.

The main contribution of the manuscript includes the following aspects:

1. In the dataset we found, pixel distribution pattern of several cancerous and healthy bone images is very similar. Due to which classification task is difficult. Therefore, after several experiments, a best feature set is identified that can classify them with high precision and accuracy even on a small dataset
2. A comparative study on selected feature set is performed with two well-known machine learning algorithm SVM and Random forest. We found SVM works best for diagnosis of human bone
3. The proposed method is more sensitive towards cancerous bone. Hence, it can be used in real time to provide second opinion to a doctor

The remaining part of the paper is organized as follows: Section 2 describes the literature survey part of the manuscript.  Section 3 defines the proposed method in detail.  Section 4 explains the result section of the proposed method.  Section 5 defines the discussion section of the proposed result. Finally, Section 6 concludes the manuscript.

## 2. Literature Survey

Avula et al. (2014) [6] proposed a strategy to distinguish the bone malignant growth from MR images utilizing mean pixel power. Ranjitha et al. (2019) [7] utilized MRI image to distinguish malignant and benign. For this, they extracted texture features and applied *K*-means clustering algorithm to separate the tumor part. From the removed tumor part, all out number of the pixel is figured, and the total number of the pixel power is determined for the extrication of the tumor part to ascertain the mean pixel value. The mean pixel value is determined to recognize malignant growth. On the off chance that the mean pixel value worth is over the limit esteem, it is considered as malignancy.

The strategy proposed by Jose et al. (2014) [8] is another methodology for brain tumor segmentation. Their strategy utilizes fuzzy *C*-means and *K*-means algorithms. In another paper presented by Patel and Doshi (2014), a noble approach is presented which can be connected utilizing diverse division methods on MRI and CT images. Reddy et al. (2015) [9] proposed a novel methodology to distinguish the size of the tumor and the bone malignancy stage utilizing developed area calculation. This strategy fragmented the district of enthusiasm by utilizing the area-developed calculation. The tumor size is determined by the number of pixels in the extricated tumor part. The contingent on the absolute pixel esteem malignant growth stage is recognized. Determination of seed point relies upon the picture, and it is hard to choose precisely.

Reddy et al. (2016) [9] have used an MRI image to detect bone cancer and stage. The image is denoised to remove noise by forming clusters based on the pixel characteristics. The value 245 and mean pixel intensity are used to predict the cancer stage. ROI (region of interest) is extracted from the image and compared with a threshold value to predict the size of the tumor. Similarly, Kaushik and Sharma (2016) [10] proposed a strategy for volume computation of disease tumors. Their methodology can be utilized in the cancerous region developing a strategy for sectioning ROI that can figure out the volume of the tumor. Sinthia and Sujatha (2016) [11] proposed a novel way to deal with the identification of the bone malignant growth utilizing the *K*-means clustering algorithm and edge recognition strategy. This strategy utilized Sobel edge identification to distinguish the edge. The Sobel edge locator identifies just the outskirt pixels. *K*-Means grouping calculation is utilized to distinguish the tumor zone.

In the same manner, Asuntha et al. (2017) [12] have developed a technique to detect bone cancer in MRI images using medical image processing techniques. The proposed method preprocessing techniques uses the Gabor filter to smooth the image and remove the noise from an image. The segmentation is carried out by using superpixel segmentation and multilevel segmentation. After filtering, edge detection and morphological operations are applied. In the second stage, superpixel segmentation is performed, and some of the important features are extracted from the images [13]. Then, the extracted features are used to identify the bone cancer. The ongoing investigation on fundamental remedial methodologies is done by Shafat et al. (2017) [14]. This paper attempts to coordinate the end of dangerous stem or forebear cells. These examinations have demonstrated that focusing on anomalies of the BM may have esteem. Their methodologies can obtain the capacity to multiply and separate novel remedial methodologies for the cutting-edge issues.

Asuntha and Srinivasan (2018) [5] stated that bone cancer is a serious disease causing the deaths of many individuals. The detection and classification system must be available to diagnose cancer at its early stage. Early detection seems to be the only factor that increases the chance of survival of cancer-affected patients. Cancer classification is a difficult and challenging task in clinical diagnosis. This paper deals with the system which uses image processing techniques to detect the tumor and classify cancer. The approach has drastically reduced the time required for the detection and classification of cancer. Nisthula and Yadhu (2013) [15] applied image enhancement techniques to increase the intensity of the image to find an edge in the cancer image. The edge detection technique has been applied. The model in this paper is designed in such a way that can detect fast and reliable cancerous tissue in the bone. Torki (2019) [16] reported tumor as one of the significant medical issues. They have developed a bone disease recognition framework. It can anticipate the malignant growth in the prior satiate. Their forecast framework is examined utilizing MATLAB-based exploratory arrangement and execution.

Vandana et al. (2020) [17] have worked on the basic bone tumor. They have upgraded the graph cut-based clustering algorithm for the identification of the cancerous part and the healthy part. Their method can be utilized to measure the attributes of danger and characterize them as typical, amiable, and malignant by utilizing multiclass irregular texture.

In the recent survey, Shrivastava et al. (2020) [18] have gone through various techniques to classify the cancerous and the healthy bone. In this work, bone computed tomography (CT) dataset in Digital Imaging and Communication in Medicine (DICOM) format are used. This work explains distinctive AI methods for tumor recognition and order. AI is an immense area of research, out of which medical image processing is a critical territory of work. In medicinal analysis like ulcer, break, tumor, and so forth image processing made the work simpler in finding the specific reason and most ideal arrangement. AI strategies are applied to restorative pictures for irregularity discovery. It can be seen that an acceptable degree of progress has been accomplished by applying the machine learning procedures. In this work, diverse AI methods for clustering are explained.

The method discussed above utilizes the segmentation techniques to obtain ROI. After that, texture and shape features are extracted to train the model. The performance of the model can be improved by selection of correct features and utilizing different types of feature optimization techniques [19, 20]. In the proposed work, different texture and shape features have been selected through rigorous experiments. These features are capable to distinguish the healthy and cancerous bone with high accuracy.

The above survey leads the work on bone cancer detection in a manner that if the feature extraction is done to get the right segmentation and finding the core part of the bone because the cancerous bone identification requires to identify all those features which are responsible for the bone cancer like bone density, bone color, and bone texture. To get the right feature, there is a need to apply the machine learning technique that can find the features and classify the healthy bone and cancerous bone. In the present research, first, we compared the efficiency of segmentation techniques like Canny, Prewitt, and Sobel to find ROI. Second, the two feature set {HOG, Entropy, Energy, Gini Index, Skewness, Contrast, Correlation, Homogeneity Product of E(X) and D(X)} and {Entropy, Energy, Gini Index, Skewness, Contrast, Correlation, Homogeneity Product of E(X) and D(X)} are prepared to train the models. Finally, we compared the performance of the Random forest and SVM using these features. The feature set {HOG, Entropy, Energy, Gini Index, Skewness, Contrast, Correlation, Homogeneity Product of E(X) and D(X)} used by the SVM provides better results compared to Random forest [21].

## 3. Material and Methods

The proposed approach flow diagram is shown in Figure 1. The input to the system is an X-ray image. The X-ray image diagnosis is fast and the cost is less.

### 3.1. Preprocessing

The X-ray image contains noise, which is removed by a median filter of the size 3 × 3. The image is blurred. Therefore, the image is sharpened to increase the intensity of the image.

#### 3.1.1. Image Segmentation

After preprocessing, the identification of an object from the image is done by segmentation. The segmentation technique's reliability is calculated based on the final precision rate. Therefore, it is rational and an effective technique for the identification of concern object. The image is parted into pixel set to gather information from the item concerned utilizing the segmentation technique (Asuntha and Srinivasan, 2018) [5]. The Canny algorithm is used to segment the image in the present research. Since, the sharp edges responsible for better ROI are obtained through the Canny edge detection algorithm [22], compared to other edge detection techniques like Sobel and Prewitt. Also, the dataset used in the study is small. The performance of the Canny edge becomes excessive as the size of the dataset increases [2, 23, 24].  Figure 2 shows the different categories of images.

#### 3.1.2. Feature Extraction

Haralick et al. [25] recommended texture descriptor is exceptionally regular to characterize texture qualities. In the Haralick descriptor, a specific pair of pixel events is determined by every section (*i*, *j*) of the GLCM matrix *A*. From the dark level estimations of the fragmented picture, we have calculated four texture features contrast, correlation, energy, and homogeneity.

Contrast: represents to the extent of neighborhood reduce level arrangement in an image and is constrained by the separation between max force and min control.

(1) $$\begin{array}{c} \text{CONT}=\underset{i,j}{\sum }{\left|i-j\right|}^{2}A_{ij}. \end{array}$$

Correlation: it measures how the pixel is coidentified with one another in the entire picture.

(2) $$\begin{array}{c} \text{CORR}=\underset{i,j}{\sum }\frac{\left(i-\mu_{i}\right)\left(j-\mu_{j}\right)A_{ij}}{\sigma_{i}\sigma_{j}}, \end{array}$$

where *μ* is the mean pixel value and *σ* is the standard deviation.

Energy: it is controlled by the summation of squared parts.

(3) $$\begin{array}{c} E=\underset{i,j}{\sum }{\left(A_{ij}\right)}^{2}. \end{array}$$

Homogeneity: it gauges the smoothness of diminished level scattering of segments; it is oppositely related to a distinction.

(4) $$\begin{array}{c} H=\underset{i,j}{\sum }\frac{A_{ij}}{1+\left|i-j\right|}. \end{array}$$

Skewness: it measures the level of turning in an image from standard scattering. The range for the allocations of the pixel is evaluated by 0 and -1 to +1.

(5) $$\begin{array}{c} \text{SK}=\sum \frac{\left({\left(\text{GLs}-\mu_{\text{GL}}\right)}^{3}*\text{PixelCount}\right)}{{\left(\text{NumberOfPixels}-1\right)}^{3}*\sigma^{3}}, \end{array}$$

where *μ* is the mean of *y*, *σ* is the standard deviation, and *X*(*t*) is the expected value of the quantity *t*. The skewness work is utilized to figure the populace's esteem.

The skewness is settled not just by what number of server farms is to the opposite side and left of the mode yet, in like manner, the detachment away they are. So, more spotlights that are on the left now near the mode may not overpower a few spotlights that are on the advantage yet altogether progressively remote away, giving a general positive skewness despite the way that more spotlights are on the left.

Variance: the variance is defined as follows.

(6) $$\begin{array}{c} \text{Var}=\frac{1}{n}\overset{n}{\underset{i=1}{\sum }}{\left|X_{i}-\mu \right|}^{2}, \end{array}$$

where *μ* is the mean of *X*:

(7) $$\begin{array}{c} \mu =\frac{1}{n}\overset{n}{\underset{i=1}{\sum }}X_{i}. \end{array}$$

Standard deviation: the standard deviation is the square root of the variance defined as follows.

(8) $$\begin{array}{c} \text{Std}=\sqrt{\frac{1}{n}\overset{n}{\underset{i=1}{\sum }}{\left|X_{i}-\mu \right|}^{2}}, \end{array}$$

where *μ* is the mean of *X*:

(9) $$\begin{array}{c} \mu =\frac{1}{n}\overset{n}{\underset{i=1}{\sum }}X_{i}. \end{array}$$

Entropy: the division of malignant growth bone is a very problematic assignment. The balanced Shannon entropy is used to perform division. Shannon entropy has been used by various pros to deal with such kinds of issues. The image is resized to 70 × 70 pixels reliant on many getting ready and test results. By then, it is turned to 35 degrees.

(10) $$\begin{array}{c} E\left(X\right)=E\left(I\left(X\right)\right)=\underset{X}{\sum }p_{y}I\left(X\right)=-\underset{X}{\sum }p_{y}\log_{2}p_{y}, \end{array}$$

(11) p=ykym1.m2,

where *k*_*y*_ is the frequency of color *x*, *m*_1_ and *m*_2_ are the total number of rows and column of the image, respectively. The force of cancer areas of bone is low. On the opposite side of the cancer bone image, entropy is high. To demand, this distinction entropy is increased by the standard deviation.

(12) $$\begin{array}{c} D\left(X\right)=E\left(I\left(X\right)\right)=\underset{X}{\sum }p_{y}I\left(X\right)*\partial \left(X\right)=-\underset{X}{\sum }p_{y}\log_{2}p_{y}*\partial \left(X\right). \end{array}$$

#### 3.1.3. Income Inequality Metrics

Income inequality metrics are utilized to gauge salary disparity and the circulation of pay in the region of financial aspects. In the present research, the Hough change aggregator grid is considered as a salary. A long queue at a predetermined edge in picture example speaks to a high salary. High-quality dissemination in the Hough collector framework speaks to inconsistent surface examples. The imbalance is calculated using the Gini index (GI) [17]. It is determined as follows.

(13) $$\begin{array}{c} \text{Gini}\_\text{Index}=\frac{2\sum_{i=1}^{n}{iX}_{i}}{n\sum_{i=1}^{n}X_{i}}-\frac{n+1}{n}, \end{array}$$

where *N* is the total number of pixels.

The estimation of the Gini index expands some spots in the extent of 0 and 1. Aggregator cross-section having corresponding distribution would yield GI respect approx. to 0 and the best clashing dispersing would yield GI worth near 1.  Figure 3 shows the feature extraction model of cancerous detection.

### 3.2. SVM Model

Bone cancer detection and classification have been carried out by SVM. A binary class classification problem uses linear SVM whereas a multiclass problem uses a multiclass SVM model. In the proposed research, linear SVM has been used for the cancerous bone and the healthy bone classification.

Let *x* be a vector denoting sample to be classified and *y* is scalar denoting their respective class label.

If ({(*p*_*i*,_*q*_*i*_), *i* = 1, 2, 3, 4..⋯*n*}) represents cancer and healthy training data. Then, *F*(*x*) decision function is constructed by SVM to correctly classify input data sets.

New pattern *p* ∈ *R*^*d*^, where the corresponding classes after classification are denoted by*y* ∈ {±1}.

The hyperplane is used to separate the classes, and it is represented as follows:

(14) $$\begin{array}{c} <u.p+b>=0,\text{and }u\in R^{d},<u.p>\text{is the inner dot product of }u\text{ and }b\text{ is a real number}. \end{array}$$

The two hyperplanes are defined by

(15) $$\begin{array}{c} u.p+b=+1,\text{when }q_{i}=\pm 1\text{ and }u.p+b=-1\text{ when }q_{i}=-1. \end{array}$$

In the present study, linear kernel function with soft margin, 1 is considered. To maximize the distance between hyperplanes equation is given by *q*_*i*_(*p*_*i*_−*u*) ≥ ±1.

#### 3.2.1. Training of SVM Model

In the proposed work, the SVM model is trained with two types of features vector. In the first experiment feature set of {HOG, Entropy, Energy, Gini Index, Skewness, Contrast, Correlation, Homogeneity Product of E(X) and D(X)} whereas, for the second experiment {Entropy, Energy, Gini Index, Skewness, Contrast, Correlation, Homogeneity Product of E(X) and D(X)} is used as a feature vector. For both, the experiment model is trained using a linear kernel with an initial learning rate of 0.001.

The hyperplane for the dataset of the proposed model is shown in Figure 4. This plane is plotted using values obtained from the features vector {Entropy, Energy, Gini Index, Skewness, Contrast, Correlation, Homogeneity Product of E(X) and D(X)}. The leaner kernel SVM model produces 8 support vectors to distinguish cancerous and healthy bone.

### 3.3. Random Forest

Random forests are an ensemble learning classification process, a regression that operates by constructing multinode decision trees while evaluating, and class mode or mean estimate of forests. The random forest algorithm extends the usual technique of aggregating bagging or bootstrap to tree learners. Instead of a training set *x* = *x*_1,_*x*_2_, ⋯*x*_*n*_ with labels *y* = *y*_1_, *y*_2,⋯_*y*_*n*_ regularly using (100 times) chooses a casual sample to supplement the set of training data and compares to these components. For *b* = 1, ⋯100.

Let *R*_*b*_(*x*) be the class prediction of the *b*th random-forest tree. Then

(16) $$\begin{array}{c} R_{1}^{100}\left(x\right)=\text{Majority}\_\text{vote}{\left\{R_{b}\left(x\right)\right\}}_{1}^{100}. \end{array}$$

## 4. Results

In the proposed work, we have performed two experiments one with hog feature sets and another without hog feature is applied on two machine learning models, i.e., random forest and SVM. Also, the performance of the models is evaluated using 5-fold cross-validation.

### 4.1. Data Set

The publicly available data sets for research on the bone X-ray image are collected from different sources such as the Indian Institute of Engineering Science and Technology, Shibpur (IIEST) and The TCIA (Cancer Imaging Archive).

#### 4.1.1. Performance Evaluation

The proposed method was implemented on MATLAB 16(a), with Microsoft Window 8 operating system and 16 GB RAM. The training dataset contains 65 images, and test dataset contains 40 images. The X-ray image contains noise, since images are collected from different sources, so it is necessary to remove the noise. The noise is removed by applying a suitable median filter of 3 × 3 sizes. The bone image is segmented by the Canny edge detection technique. The features are extracted from the cancerous and the healthy image. The training and classification are performed using SVM. The symmetrical or asymmetrical distribution of pixels in the image is measured by the skewness. The skewness of the cancerous bone is less compared to the healthy bone due to the asymmetrical distribution of pixels in the cancerous bone.

The training image =∑_*i*=1_^65^*C*_*i*_.

where *i* = 1 to 45, we consider cancerous bone image and *i* = 46 to 65 healthy bone images. The skewness value in the training image is shown in Figure 5. The skewness value of the test image is shown in Figure 6. The pattern of skewness value in the cancerous and the healthy bone is similar in the test and training image.

#### 4.1.2. Performance Evaluation with HOG Feature

The HOG feature plays a vital role in training and classification. It gives shape as well as the direction of a pixel in the image by extracting gradient and orientation. The HOG descriptor divides the image into smaller regions, and for each region, the histogram is generated. First, the image is resized to 25 × 25 pixels sizes. The window size per bounding box is set to 3, and the number of histogram bins is set to 6 after several experiments on the data set. The gradient in the *x* and *y* direction is calculated for every pixel to check the change in intensity of the image. The test result of the data set with the HOG feature is shown in Figure 7. Out of 20 cancerous bones, 1 is false-negative, and out of 20 healthy bone images, 2 are false positive. In Figure 8, the hog feature has not been applied for training and testing of the data set due to which out of 20 cancerous bones, 2 are false-negative, and out of 20 healthy bones, 3 are false positive.

The confusion matrix of test data with hog feature and without hog feature has been shown in Tables 1 and 2.

The comparison of test data based on accuracy, precession, recall, and *F*1 score is shown in Table 3.

From Table 3, it can be suggested that hog is one of the important features for the identification and classification of healthy and cancerous bone. Similar researches have used GLCM-based texture features and other texture features for the identification and classification of healthy and cancerous bone.

### 4.2. Performance Evaluation Using 5-Fold Cross-Validation

The dataset used in the study contains 105 images out of which 65 are bone cancer and 40 are healthy bone. To avoid bias performance measures of the proposed model, we have applied 5-fold cross-validation on the data set. The confusion matrices of the Random forest and SVM model are shown in Figures 9 and 10.

The training and validation loss curve of the proposed model is shown in Figure 11. Due to the small dataset, the loss curve is not saturated. We can see that the maximum loss is less than 1. This loss can be further reduced by training for more epochs on large dataset.

### 4.3. Box Plot Analysis

To find the importance of the features, the box plot analysis is also performed.  Figure 12 represents the box plot of the 9 features. The hog feature is represented by the ninth box plot in Figure 12, and the parallel box plot is a representation of all the features. The data of the HOG feature contains the data in a smooth form, and there is no fluctuation in the data therefore the classification is done using HOG is accurate, as compared to other features. It gives shape as well as the direction of a pixel in the image by extracting gradient and orientation. The HOG descriptor divides the image into smaller regions, and for each region, the histogram is generated. The gradient in the *x* and *y* direction is calculated for every pixel to check the change in intensity of the image.

## 5. Discussion

Bone cancer is growing day by day researches reported that it happens due to fluid, fat cells, and hematopoietic cells. This differentiation can be identified using texture analysis. The texture is represented by the intensity of the pixels. The intensity of the pixels in the healthy and the cancerous bone is different. Therefore, using texture features classification of the image can be performed. The texture of the cancerous and healthy bone is different. So, it is necessary to correctly identify texture (Reischauer et al., 2018) [26].

The healthy bone pixels are less scattered as compared to the cancerous region. The research of Reddy et al. (2016) [27] has used the mean pixel to segment the cancerous bone. But the classification of the bone image into the healthy and cancerous is not performed. The method calculated ROI (region of interest) from cancerous affected MRI bone image. The affected area's analysis is performed based on the number of pixels. After that, the mean intensity is calculated by the sum of the intensity of the pixel extracted. Finally, based on the mean intensity value, cancer stage is predicted. The research of Asuntha et al. (2017) [12] has used GLCM-based texture features to identify the cancerous bone. The research is not able to classify the bone into respective category.

The GLCM texture feature alone is not sufficient for bone cancer classification. Therefore, in the present research apart from the basic four texture features of the GLCM, other features like the hog have been used to identify and classify the cancerous bones. The hog feature gives the shape and direction of the pixels in the images on local cells. The hog featured can identify the cancerous region. In the paper of Bandyopadhyay et al. (2018) [2] has used a fusion of several techniques and texture features to identify and classify the cancerous bone and the healthy bone. The classification of the long bone is performed using SVM. The method is focused only on the long healthy and cancerous bone. The performance of models is 85%, which can be further improved. The present study is not only limited to the long bone.

### 5.1. Comparison of the Machine Learning Algorithms

The present study compared the potential of the machine learning algorithm, i.e., SVM and Random forest on the selected feature using 5-fold cross-validation scheme, shown in Table 4. The features for machine learning are not changed during training.

In all the measurement parameters, SVM is better than random forest machine learning. Therefore, in the present study, SVM has been chosen for the diagnosis of cancerous and healthy bone.

The cancerous region pixels are more scattered in the bone image (Oishila et al., 2018) [2]. The HOG feature calculates the shape and direction of pixels based on window size and the histogram bins. The ROI is extracted by a bounding box and the largest contour region, as shown in Figure 13.

### 5.2. Comparison of the Proposed Approach with Previous Work

The proposed approach has been compared with the existing approach (Oishila et al., 2018) [2] based on texture features such as entropy, standard deviation. The existing approach could not lead the solutions for different types of human bone like flat bone and irregular bone. The proposed approach is using hog features along with entropy and standard deviation to identify the cancerous and the healthy bone for the different types of human bone. The proposed approach is better in terms of all the parameters. The *F*1-score of the proposed model, 0.94 is better than the *F*1-score 0.88 of the work [2] for cancerous bone classification.  Table 5 shows the comparison of the present approach with the existing work.

The graphical representation of the proposed work with previous work is shown in Figure 14. The SVM model with hog feature set outperforms for all measures compared to work [2] without 5-fold cross-validation. With 5-fold cross-validation performance measure like accuracy and recall is much higher than work [2] but precision and *F*1-score are slightly less than the work [2].

## 6. Conclusion

The proposed method is a combination of feature extraction and classification model that discriminate vitality of the cancerous and healthy bone identification and classification. The median filter of size 3 × 3 is used to remove the noise. The object of interest is extracted by applying the canny algorithm. The textures of the cancerous and healthy bone are different in the cancerous region. In the cancerous region, the pixel of the cancerous bone is more scattered compared to the healthy bone. Therefore, it is important to select the texture feature which can differentiate cancerous region. The most appropriate texture feature used by researchers is the GLCM-based texture feature. But it found in the experiment that only GLCM-based texture feature is not sufficient. The entropy and skewness also play a vital role in cancerous region prediction. The value of entropy is low in the cancerous region and high outside the cancerous region. The hog feature gives the shape and direction of a pixel in images. The experiment found that using the hog feature with the GLCM texture feature gives an *F*1-score of 92.68%, better than without using the hog feature of 87.80%. According to the ground truth, the accuracy of 92.30% with hog features is obtained, which is better than previous work (Oishila et al., 2018) [2] of 85% for cancerous bone. The performance of the system can be further improved by selecting other texture features. In short, we can summarize, and proposed method can detect cancerous and healthy bone image with high precision. Our model performance is more sensitive towards cancers bone image compared to healthy bone image. That indicates it can be used in real time to provide second opinion to a doctor. In the future, we will create a large dataset to further evaluate the performance of the model. We will also work on the feature optimization techniques like monarch butterfly optimization (MBO), earthworm optimization algorithm (EWA), elephant herding optimization (EHO), moth search (MS) algorithm, slime mould algorithm (SMA), and Harris hawks optimization (HHO) for improvement of performance.

## Figures and Tables

**Figure 1:** The system flow diagram of the proposed work.

**Figure 2:** Different types of images after processing.

**Figure 3:** Feature extraction model of cancerous detection.

**Figure 4:** Hyperplane of linear kernel SVM.

**Figure 5:** Skewness patterns in training data.

**Figure 6:** Skewness patterns in test data.

**Figure 7:** Test data result with the hog feature.

**Figure 8:** Test data result without hog feature.

**Figure 9:** 5-fold cross-validation confusion matrix using Random forest.

**Figure 10:** 5-fold cross-validation confusion matrix using SVM.

**Figure 11:** Training and validation loss curve of the proposed method.

**Figure 12:** Box plot analysis of different features.

**Figure 13:** Image with hog feature.

**Figure 14:** Performance measures comparison with previous work [2].

**Table 1:** Hog feature-based confusion matrix of test data.

Samples	No. of images	Cancerous	Healthy
Cancerous bone	20	19	1
Healthy bone	20	2	18

**Table 2:** Without hog feature-based confusion matrix of test data.

Samples	No. of images	Cancerous	Healthy
Cancerous bone	20	18	2
Healthy bone	20	3	17

**Table 3:** Comparisons of accuracy, precision, recall, and *F*1-score with HOG feature and without HOG features.

Measure	Without hog feature (%)	With hog feature (%)
Accuracy	87.5	92.50
Precision	85.71	90.47
Recall	90	95
*F*1 score	87.80	92.68

**Table 4:** Comparison of the machine learning algorithms.

Measure	Random forest	SVM
Accuracy	69.23	92.50
Precision	75.56	90.47
Recall	79.06	95
*F*1 score	77.27	92.68

**Table 5:** Comparison of the previous work [2] and the proposed approach for cancerous bone classification.

Measure	Previous work	The proposed approach
Accuracy	0.84	0.92
Precision	0.87	0.93
Recall	0.80	0.89
*F*1 score	0.88	0.94

## Data Availability

No data is available.
